# High Performance Computing Simulation of Intelligent Logistics Management Based on Shortest Path Algorithm

**DOI:** 10.1155/2022/7930553

**Published:** 2022-06-08

**Authors:** Zongchao Wei

**Affiliations:** Developing and Planning Department, Yellow River Conservancy Technical Institute, Kaifeng 475004, China

## Abstract

At present, e-commerce drives the logistics industry to develop greatly, but at the same time, there is a huge demand in this field, such as lower cost and higher efficiency. Facing the needs of logistics management development, it needs the blessing of intelligent technology, which involves countless fields at present. Intelligent logistics management has become a hot spot at present. What needs to be solved in this respect is how to shorten the transportation distance and save costs. To solve this problem, this paper proposes to introduce the shortest path algorithm. This paper compares the Dijkstra algorithm with the A^*∗*^ algorithm under the background of logistics management and finds that the latter is more suitable for this field with huge amount of information. In order to improve the performance of the A^*∗*^ algorithm, this paper introduces ant colony algorithm, which can better avoid obstacles. Combining these two algorithms, a ^*∗*^-ant colony algorithm is obtained. The algorithm absorbs the advantages of the two algorithms, while maintaining high efficiency and good stability. These characteristics are very satisfying in the field of logistics management. Through the performance test and simulation experiment, it is concluded that the algorithm has excellent optimization ability and can reduce the cost for this field.

## 1. Introduction

The awakening of e-commerce also awakens the development of logistics industry. At the same time, China pays great importance to logistics management. It is also the idea that the country wants to innovate and change to collide with the field of intelligent technology and logistics management. With the addition of intelligent technology, it can solve the shortest path problem well, thus reducing the cost. The shortest path algorithm is a good medicine to solve this problem. Under the test of the traditional shortest path algorithm, it is found that it can no longer meet the current problem, so it is necessary to innovate and change the algorithm. And, this is undoubtedly the mutual achievement of the two. The level of logistics management can be improved only when the two develop mutually.

In literature [1], the shortest path problem has penetrated into a wide range of fields. The Dijkstra algorithm is not perfect. First, its exit mechanism is not applicable to undirected graphs; second, the problem of adjacent nodes is a great hidden danger; third, the problems of multivertex are not fully considered. In literature [2], the *k*-shortest path algorithm also has some defects in some aspects, and the alternative path obtained by the algorithm cannot be proved to be substantially different from the original path. In reality, network extension technology is usually used to solve the problems caused by turning restriction, but this method also has defects. Therefore, researchers introduce links to improve and solve this problem. The advantage of this model is to eliminate overlapping paths and find alternative paths, which can finally reduce similarity and only rely on its own nodes and links to complete the operation. In literature [3], distributed algorithm gives the shortest path problem a shot in the arm, the most important component of which is BHC. The related problems can be solved by calculating the time complexity. For example, each node can use multiple processors and how much time complexity can be calculated through these processors, so that this kind of problem can be well solved. In literature [4], the network shortest path problem is relatively simple to solve. The fact is that a single objective function is incapable of describing problems appropriately in real life. While pursuing fast time, it may bring high cost. This is like a seesaw, but it still needs a way to balance the seesaw. The force that can balance the seesaw is Pareto. In literature [5], in the field of genes, this algorithm has also made some achievements. Dijkstra algorithm is like a good medicine to diagnose and treat gene-related problems. And, all genes in this path are candidate genes. Only a few genes were selected in the end. In literature [6], all objects have their own sizes and shapes, and researchers suggest that this algorithm has achieved little in motion planning. The idea of shape decomposition is put forward to solve this problem. Decomposition and iteration are a pair of enemies, and it is their choice to have more you and less me. Then, the geometric algorithm is the judge to judge whether there will be a war between them. If there is no hidden danger, the shortest path can be calculated by grass fire algorithm. In literature [7], researchers combine the graph algorithm with active contour restoration. Finding the global minimum is the trick of graph algorithm. Generally speaking, ordinary active contours cannot be run with three or more pixels in mind. Therefore, the researchers put forward a correct definition of deformable template and use the Dijkstra algorithm to track the contour. In literature [8], in order to study the relationship between user interface and satisfaction, the Dijkstra algorithm is used for experiments. Apple and Android are the two kings of mobile models. Students were recruited to conduct experiments on this. After testing, it was found that IOS was more useful than Android for Dijkstra algorithm. In literature [9], China has summarized all aspects of logistics. After analyzing the logistics demand, the researcher proposed to introduce relevant technical software support. For the problems related to the path, the relevant personnel and institutions decided to adopt logical data structure. In literature [10], the article agrees that intelligent technology is unshakable. Therefore, we can only find another way to change from a strategic perspective. At the same time, it shows that the addition of intelligent technology has brought many qualitative changes to this field. Compared with traditional methods, intelligent logistics application has been recognized as the best management method at present. In literature [11], the Internet of Things and cloud computing have propped up a sky, sheltering intelligent logistics from the wind and rain. In literature [12], in order to keep up with the development trend of intelligent logistics demand, it is necessary to shorten the cycle and cost while designing the system. In the whole process, there must be methods to implement both people and things. A series of technologies such as GPS have also been applied. Therefore, intelligent logistics will provide a good ascending ladder for e-commerce. In literature [13], in medical use, logistics management is also very important. Hospitals will encounter a series of problems when quoting a set of logistics management mode, which researchers need to analyze and popularize in hospitals after using the logistics management mode. At the same time, this model also needs to be improved. In this way, hospital consumables can be reduced, and costs can be reduced. In literature [14], it is recognized by most enterprises that production and transportation become one. Cost and time are important factors in the whole process. If you want to taste the sweetness, you have to give up. This price is the control of information. For logistics management, the ultimate destination must be gradually networked and then set different frameworks according to different needs. In literature [15], Internet of Things has been the backbone of logistics development, which is the development trend of the times. Researchers need to analyze and predict the architecture, which will be a historic change.

## 2. Shortest Path Algorithm

As its name implies, the shortest path algorithm is a corresponding algorithm proposed to solve the shortest path problem, and the shortest path is the path with the minimum sum of the weights of edges in the process of starting from one vertex to another in a graph.

### 2.1. Dijkstra Algorithm

Dijkstra algorithm is a classical algorithm for solving the shortest path, and the core of its algorithm is the order of the length of the path. The main purpose of this algorithm is to choose the best route in the logistics transportation nodes.

The Dijkstra algorithm flow is shown in Figure 1:

The final shortest path length *D*[*j*] is expressed as follows:

(1) $$\begin{array}{c} D\left[j\right]=\min\left\{D\left[i\right]|v_{i}\in V\right\}. \end{array}$$

*D*[*i*]: shortest path length from shipment starting point to each receiving point. *v*: logistics starting point. *v*_*i*_: end point.

After the shortest path is obtained, the shortest path length among the remaining paths is as follows:

(2) $$\begin{array}{c} D\left[j\right]=\min\left\{D\left[i\right]|v_{i}\in V-S\right\}, \end{array}$$

(3) $$\begin{array}{c} S=S\cup \left\{v_{j}\right\}. \end{array}$$

*S*: the shortest path set obtained. *v*_*j*_: the shortest path end point of the remaining path starting from *v*.

At the same time, modify the shortest path that the remaining paths can reach *v*_*k*_, and the formula is as follows:

(4) $$\begin{array}{c} D\left[k\right]=D\left[j\right]+arcs\left[j\right]\left[k\right]\text{if}D\left[j\right]+arcs\left[j\right]\left[k\right]<D\left[k\right]. \end{array}$$

### 2.2. A^*∗*^ Algorithm

The right-hand man of A^*∗*^ algorithm is not only the evaluation function but also the search direction. In the logistics system, in the process of finding the shortest path, there are 8 nodes around the starting point, and these nodes are adjacent to the starting point. With the help of his right-hand man, the node with the lowest value will soon be found out and given the search for the next extended node. Repeat the above operations, and the lowest cost path comes into being.

The A^*∗*^ algorithm flow is shown in Figure 2:

The formula of heuristic function is as follows:

(5) $$\begin{array}{c} f\left(n\right)=g\left(n\right)+h\left(n\right), \end{array}$$

(6) $$\begin{array}{c} g\left(n\right)=L_{i}+\sqrt{{\left(x_{n}-x_{i}\right)}^{2}+{\left(y_{n}-y_{i}\right)}^{2}}, \end{array}$$

(7) $$\begin{array}{c} h\left(n\right)=L_{i}+\sqrt{{\left(x_{n}-x_{T}\right)}^{2}+{\left(y_{n}-y_{T}\right)}^{2}}. \end{array}$$

*f*(*n*): cost function of node *n*. *g*(*n*): actual cost from starting point to node *n*. *h*(*n*): estimated cost of node *n* to the end point. *x*_*n*_ ′*y*_*n*_: horizontal and ordinate values of node *n*. *x*_*i*_ ′*y*_*i*_: horizontal and ordinate values of current node *i*. *x*_*T*_ ′*y*_*T*_: horizontal and ordinate values of the end point. *L*_*i*_: actual cost from the starting point to the current node *i*.

## 3. Optimization Algorithm

In logistics management, the above two algorithms can speed up this field. But even in terms of legal skills, there is still a gap between the two. When the digraph using Dijkstra algorithm has *n* vertices, the complexity of the algorithm is *O*(*n*^2^). Obviously, this algorithm is very efficient in solving single source path in directed graphs with all positive weighted edges, but it cannot combine more useful information to search, which is undoubtedly a fatal blow in logistics management with huge amount of information.

A^*∗*^ algorithm has the characteristics of Dijkstra algorithm mentioned above, and A^*∗*^ algorithm can maintain stability; at the same time, it has high-speed operation and accurate results. It can be seen from this that A^*∗*^ algorithm is more efficient in logistics management. But the A^*∗*^ algorithm still needs to be improved.

### 3.1. Improved A^*∗*^ Algorithm

#### 3.1.1. Improved Node

There are *n* nodes in a single road section, and the search efficiency for *n* nodes one by one is too low, so this paper proposes to extract only the beginning and end nodes in a single road section, which greatly improves the search efficiency. Specific improvements are shown in Figure 3:

#### 3.1.2. Improved Database

Logistics transportation usually takes each transfer point as a unit, and the amount of data in the network database of each transfer point is huge. General logistics management is to use direct reading means for data, but this is inefficient. Therefore, this paper puts forward the combination of database and memory and stores it in batches according to time. In this way, data can be obtained from the cache, thus greatly improving the efficiency of data query and search.

#### 3.1.3. Improved Heuristic Function

In this paper, the evaluation standard of the evaluation function is travel time, while the heuristic function can be determined by the ratio of the distance between two nodes to the logistics speed. The formula of travel time estimation *h*(*n*) is as follows:

(8) $$\begin{array}{c} h\left(n\right)=\frac{d\left(n,e\right)}{\bar{v}}, \end{array}$$

(9) $$\begin{array}{c} d\left(n,e\right)=R\times \;\arccos\left[\cos\left(\frac{\pi x_{n}}{180}-\frac{\pi x_{e}}{180}\right)\cos\frac{\pi y_{n}}{180}\cos\frac{\pi y_{e}}{180}+\sin\frac{\pi y_{n}}{180}\sin\frac{\pi y_{e}}{180}\right], \end{array}$$

(10) $$\begin{array}{c} \bar{v}=\frac{1}{m}\sum_{i=1}^{m}v_{i}. \end{array}$$

*d*(*n*, *e*): actual distance between node *n* and target node *e*. $\bar{v}$: average vehicle speed. R: radius of the Earth, with the value of. 6.37 × 10^6^*m*. *v*_*i*_: speed on road section *i*. *m*: the range involved in the formula is the total number of road sections in the logistics area.

### 3.2. Ant Colony Algorithm

The core content of the algorithm, Ant *k*, judges the choice path by pheromones and leaves pheromones for stacking. Finally, we can get the shortest path. The flow chart of ant colony algorithm is shown in Figure 4:

At first, when *τ*_ij_(0)=*τ*^0^, this means that ants do not understand the environment, and they need to determine the path by the transition probability *P*_*ij*_^*k*^(*t*) from node *i* to *j*. The transition probability *P*_*ij*_^*k*^(*t*) is expressed as follows:

(11) $$\begin{array}{c} P_{ij}^{k}\left(t\right)=\left\{\begin{array}{cc} \frac{{\left[\tau_{ij}\left(t\right)\right]}^{\alpha }\cdot {\left[\eta_{ij}\left(t\right)\right]}^{\beta }}{\sum {\left[\tau_{ij}\left(t\right)\right]}^{\alpha }\cdot {\left[\eta_{ij}\left(t\right)\right]}^{\beta }}, & j\in a_{k},\\ 0, & j\notin a_{k}, \end{array}\right. \end{array}$$

(12) $$\begin{array}{c} \eta_{ij}=\frac{1}{d_{ij}}. \end{array}$$

*τ*_ij_(*t*): the pheromone left by ant *k* on path *i*, *j* at time *t*. *η*_ij_(*t*): distance heuristic factor. *d*_*ij*_: distance between nodes *i* and *j*. *α*: relatively important factors about ant information trajectory. *β*: relative importance factor of heuristic function. *a*_*k*_: a set of nodes to which goods *k* in the logistics are allowed to arrive next.

After ants move for a long time, pheromones remaining in the path will volatilize like alcohol. Therefore, the pheromone on the path should be updated after each cycle of ants. The pheromone update formula is as follows:

(13) $$\begin{array}{c} \tau_{ij}\left(t+1\right)=\rho \tau_{ij}\left(t\right)+\Delta \tau_{ij}\left(t,t+1\right), \end{array}$$

(14) $$\begin{array}{c} \Delta \tau_{ij}\left(t,t+1\right)=\sum_{k=1}^{m}\Delta \tau_{ij}^{k}\left(t,t+1\right). \end{array}$$

*ρ*: pheromone volatilization coefficient. Δ*τ*_*ij*_^*k*^: pheromones left by ant *k* on paths *i* and *j*. Δ*τ*_*ij*_: pheromone increment left by ants on paths *i* and *j*.

The three formulas for Δ*τ*_*ij*_ are as follows:

(15) $$\begin{array}{c} \Delta \tau_{ij}^{k}\left(t,t+1\right)=\frac{C}{L_{k}}, \end{array}$$

(16) $$\begin{array}{c} \Delta \tau_{ij}^{k}\left(t,t+1\right)=\frac{C}{d_{ij}}, \end{array}$$

(17) $$\begin{array}{c} \Delta \tau_{ij}^{k}\left(t,t+1\right)=C. \end{array}$$

*L*_*k*_: path length of ant *k* once cycle. C: constant.

### 3.3. A^*∗*^-Ant Colony Algorithm

A^*∗*^-ant colony algorithm for logistics path planning is divided into global and local. The initial global planning is to use A^*∗*^ algorithm to calculate, with the passage of time to search for complex environment, the planning problems encountered by ant colony algorithm, which can effectively avoid obstacles and avoid local deadlock. The algorithm flow is shown in Figure 5:

#### 3.3.1. Node Selection and Information Update

However, ant colony algorithm also has some defects, such as the global search ability is not strong, convergence speed is not high, and a series of problems. This will make the whole algorithm appear a series of cases such as local optimum. Therefore, it is necessary to further improve the ant colony algorithm before it can be merged with A^*∗*^ algorithm to obtain A^*∗*^-ant colony hybrid algorithm.

Assuming that there are *m* goods to be transported by logistics in this area, the formula for *m* is as follows:

(18) $$\begin{array}{c} m=\sum_{i=1}^{n}b_{i}\left(t\right), \end{array}$$

*n*: total number of target nodes in this area. *b*_*i*_(*t*): quantity of logistics goods at node *i* at time *t*.

The formula for the probability of goods *k* transported by logistics moving from node *i* to node *j* is as follows:

(19) $$\begin{array}{c} j=\left\{\begin{array}{cc} \max\left\{\tau_{iS}^{\alpha }\left(t\right)\eta_{iS}^{\beta }\left(t\right)\right\}, & S\in a_{k},r>\rho_{0},\\ \text{choose }j\text{ according to }p_{ij}^{k}\left(t\right), & \text{otherwise,} \end{array}\right. \end{array}$$

(20) $$\begin{array}{c} P_{ij}^{k}\left(t\right)=\left\{\begin{array}{cc} \frac{\tau_{ij}^{\alpha }\left(t\right)\eta_{ij}^{\beta }\left(t\right)}{\sum_{S\in a_{k}}\tau_{ij}^{\alpha }\left(t\right)\eta_{ij}^{\beta }\left(t\right)}, & j\in a_{k},\\ 0, & \text{others,} \end{array}\right. \end{array}$$

max{*τ*_*iS*_^*α*^(*t*)*η*_*iS*_^*β*^(*t*)}: the node of the path with the largest amount of information in the path set related to the node *i*.

When the whole iteration is completed, the best path, that is, the shortest path, will be selected, and the pheromones of each node on this path will be updated. The updated formula is as follows:

(21) $$\begin{array}{c} \tau_{ij}\left(t+1\right)=\left(1-\rho \right)\tau_{ij}\left(t\right)+\rho \Delta \tau_{ij}\left(t,t+1\right), \end{array}$$

(22) $$\begin{array}{c} \Delta \tau_{ij}\left(t,t+1\right)=\frac{1}{L_{l}}. \end{array}$$

*L*_*l*_: the optimal path length of the whole search in this iteration.

## 4. Simulation Experiment

### 4.1. Algorithm Testing

#### 4.1.1. Parameters and Environment Settings

In this test, the grid method is adopted, and 10^*∗*^10 grids are divided, in which the white grid represents the logistics transportation area and the black grid represents the obstacles. Set the ant size to 50 and the maximum iteration number to 100.

*α*=1, *β*=5 , *ρ*=0.7 , *τ*_0_=4,  and   *Q*=2000 for Dijkstra algorithm, A^*∗*^ algorithm, and A^*∗*^-ant colony algorithm for path planning and experiment. The experimental results of Dijkstra algorithm are shown in Figure 6:

The experimental results of A^*∗*^ algorithm are shown in Figure 7:

The experimental results of A^*∗*^-ant colony algorithm are shown in Figure 8:

The length and running time data of the path are shown in Table 1:

As can be seen from the above chart, for these three algorithms, in terms of time, A^*∗*^ algorithm has the shortest running time and the fastest search speed. But from the shortest path point of view, the shortest path found by the algorithm proposed in this paper is better. From the combination of these two aspects, it can be concluded that the advantages of the A^*∗*^-ant colony algorithm are not particularly prominent in the simulation environment, but the overall performance is still due to the other two. For the logistics management environment, the A^*∗*^-ant colony algorithm can better play its advantages. For such a large environment as logistics management, there are much more nodes to search than tests. With iterative updating, the A^*∗*^-ant colony algorithm can give full play to its advantages, while the first two algorithms are not suitable for such a large amount of data operations.

### 4.2. Simulation Experiment

#### 4.2.1. Establishment of an Objective Function

This experiment will compare the three algorithms from the path length, cost, and speed.

The formula of the minimum cost is as follows:

(23) $$\begin{array}{c} F_{i}=\sum_{j\in J}C_{ij}X_{ij}+f_{ki}\;i\in I, \end{array}$$

(24) $$\begin{array}{c} \min F^{\prime }=\sum_{k=1}^{q}\sum_{j=1}^{n}C_{kj}X_{kj}, \end{array}$$

(25) $$\begin{array}{c} \sum_{j=1}^{n}X_{kj}\leq d_{k}, \end{array}$$

(26) $$\begin{array}{c} \sum_{k=1}^{q}X_{kj}\geq b_{j}. \end{array}$$

*F*_*i*_: cost of transportation from node *i*. *C*_*ij*_: management fee of goods transported from node *i* required by user *j*. *X*_*ij*_: the quantity of goods transported from the node *i* required by the user *j*. *C*_*kj*_: management fee of goods at outlet *k* required by user *j*. *X*_*ij*_: the quantity of goods from the outlet *k* required by the user *j*. *f*_*ki*_: the cost of setting the dot *k* in the experimental delimited area. *d*_*k*_`*b*_*j*_: maximum setting size of outlets and demand of users *j*.

#### 4.2.2. Simulation Results and Experimental Analysis

Set a certain area as logistics transportation area and transform it into a 50^*∗*^50 grid range. Suppose it needs to be delivered to 10 users for 10 times, and there are 8 outlets in total. Three algorithms are used to predict the shortest path length, find the shortest path time and transportation cost of these 10 times, and compare with the actual values.

The shortest path length data obtained through experiments are shown in Table 2:

The experimental data of finding the shortest path time are shown in Table 3.

The transportation cost data obtained through experiments are shown in Table 4.

The algorithm for the shortest path pair is shown in Figure 9.

The algorithm pair finds the shortest path time pair as shown in Figure 10.

The algorithm for transportation cost pairs is shown in Figure 11.

It can be seen from the above icon that, in terms of finding the shortest path and transportation cost, it is obvious that the algorithm proposed in this paper can better calculate and find the shortest path, which shows that the algorithm has been improved and greatly improved the optimization ability. In terms of running time, we can see that, in the early stage of running, the speed of the A^*∗*^ algorithm is still relatively fast, but with the increase of iteration times, the increasing number of nodes, and the continuous accumulation of information, the speed of A^*∗*^ algorithm cannot be well maintained, while the algorithm proposed in this paper is more consistent with the data in the later stage.

## 5. Conclusion

For the Dijkstra algorithm, facing a large amount of information, it does not have the ability to use it reasonably, which makes it and A^*∗*^ algorithm have a gap in logistics and transportation. This is also one of the reasons for choosing the A^*∗*^ algorithm in this paper. A^*∗*^ algorithm is really excellent in terms of running speed, but in terms of logistics and transportation, the algorithm proposed in this paper can provide stable development for later operation. At the same time, it can be found from the experiment that the performance of the algorithm is stable, and the high stability and accuracy can be combined with logistics and transportation. The logistics management in the future tends to be more intelligent, and the intelligent technology is constantly developing, which is a further excavation assistant for intelligent logistics management.

## Figures and Tables

**Figure 1:** Flow chart of Dijkstra algorithm.

**Figure 2:** A^∗^ algorithm flow chart.

**Figure 3:** Node improvement diagram.

**Figure 4:** Flow chart of the ant colony algorithm.

**Figure 5:** A∗-ant colony algorithm diagram.

**Figure 6:** Dijkstra algorithm simulation path diagram.

**Figure 7:** A∗ algorithm simulation path diagram.

**Figure 8:** A∗-ant colony algorithm simulation path diagram.

**Figure 9:** Comparison diagram of the algorithm against shortest path.

**Figure 10:** Comparison diagram of the algorithm to find the shortest path time.

**Figure 11:** Comparison of algorithm and transportation cost.

**Table 1:** Path length and running time data table.

Algorithm	Path length	Running time
Dijkstra	16.24	7.89
A^∗^	13.99	1.32
A^∗^-ant colony algorithm	13.31	3.79

**Table 2:** Shortest path length data table.

Serial number	Dijkstra	A^*∗*^	A^*∗*^-ant colony algorithm	Actual value
1	24.5	21.3	15.3	14.1
2	30.7	25.9	20.2	21.1
3	16.9	13.2	11.4	10.2
4	22.5	20.4	13.9	13.9
5	27.9	22.4	17.8	16.9
6	10.5	8.9	5.1	6.4
7	21.1	15.6	10.2	11.3
8	11.6	8.2	4.3	4.6
9	15.4	9.3	4.8	5.1
10	20.4	13.9	10.3	10.5

**Table 3:** Data table for finding the shortest path time.

Serial number	Dijkstra	A^*∗*^	A^*∗*^-ant colony algorithm	Actual value
1	32	10	20	11
2	33	15	16	13
3	42	20	30	23
4	41	5	30	12
5	39	20	21	22
6	31	15	13	13
7	32	23	16	17
8	36	19	17	16
9	35	21	18	19
10	46	25	19	19

**Table 4:** Data sheet of transportation cost.

Serial number	Dijkstra	A^*∗*^	A^*∗*^-ant colony algorithm	Actual value
1	2.5	2.1	1.5	1.3
2	3.1	2.6	2.1	2.2
3	1.5	1.9	1.8	2.0
4	2.3	2.5	1.7	1.9
5	2.8	2.9	2.5	2.2
6	1.2	1.1	0.5	0.9
7	2.0	1.7	1.5	1.6
8	1.4	1.2	0.8	0.7
9	1.9	2.2	1.2	1.3
10	2.2	2.4	1.9	1.5

## Data Availability

The experimental data used to support the findings of this study are available from the corresponding author upon request.
